# Bioactive Compounds and Therapeutics from Fish: Revisiting Their Suitability in Functional Foods to Enhance Human Wellbeing

**DOI:** 10.1155/2022/3661866

**Published:** 2022-08-05

**Authors:** Chinaza Godswill Awuchi, Charles Nnanna Chukwu, Adams Ovie Iyiola, Sana Noreen, Sonia Morya, Ademiku O. Adeleye, Hannington Twinomuhwezi, Katarzyna Leicht, Nancy Bonareri Mitaki, Charles Odilichukwu R. Okpala

**Affiliations:** ^1^School of Natural and Applied Sciences, Kampala International University, Kampala, Uganda; ^2^Department of Biochemistry, Michael Okpara University of Agriculture, Umudike, Nigeria; ^3^Department of Fisheries and Aquatic Resources Management, Osun State University, Ejigbo Campus, Osun State, Nigeria; ^4^Institute of Diet and Nutritional Sciences, University of Lahore, Lahore, Pakistan; ^5^Department of Food Technology & Nutrition, Lovely Professional University, Phagwara, 144411 Punjab, India; ^6^Faith Heroic Generation, No. 36 Temidire Street, Along Oloko Area, Azure, Ondo State, Nigeria; ^7^Department of Chemistry, Kyambogo University, Kyambogo, Uganda; ^8^Department of Functional Food Products Development, Wrocław University of Environmental and Life Sciences, 51-630 Wrocław, Poland

## Abstract

Global public awareness about fish-based diet and its health/nutritional benefits is on the rise. Fish nutritional profile projects promising bioactive and other compounds with innumerable health benefits for human wellbeing. As various reported researches involving fish/marine-derived molecules reveal promising attributes, and as the position of fish-based nutrients as nutraceuticals continue to strengthen, health challenges still confront communities worldwide, from cardiovascular disease, diabetes, and obesity to hypertension. Thus, further understanding of fish-based nutrient impact as functional foods remains crucial given the diverse prevailing compositional/nutraceutical merits. In this review, therefore, we provide important information regarding bioactive compounds and therapeutics obtained from fish, specific to the context of their suitability in functional foods to enhance human health. This contribution is hereby constructed as follows: (a) fish nutraceutical/therapeutic components, (b) constituents of fish-based nutrients and their suitability in functional foods, (c) fish antioxidant/bioactive compounds to help alleviate health conditions, (d) common human ailments alleviated by fish-based nutrients, and (e) role of fish in mental health and immune system. As increased fish consumption should be encouraged, the potential of the quality proteins, omega-3 fatty acids, and other compounds inherent in fish should steadily be harnessed.

## 1. Introduction

Global public awareness about seafood diet and its health/nutritional benefits is on the rise. Besides bioactive compounds in seafood supporting human body growth and function, therapeutic potentials therein help alleviate as well as manage disease conditions. Hence, scientists constantly explore these bioactive constituents/therapeutic potentials to improve populace health and quality of life [1, 2]. The beneficial effects of bioactive compounds happen through such physiological mechanisms as antioxidant activity, hormonal actions, and immune system enhancement to facilitate substance transit via the digestive tract, colonic butyric acid production, and (gut) absorption/dilution [3, 4]. Fish products, in addition to providing bioactive constituent of nutritional/therapeutic values that improve human wellbeing, remain conventionally cheap protein sources [5–8]. Such bioactive constituents like proteins, lipids, minerals, vitamins, and other fish by-products also possess important therapeutic potentials. together with high amounts of long-chain omega-3 polyunsaturated fatty acids (PUFAs) [1]. Bioactive constituents in fish/marine products situate as very promising alternatives over nonnatural types [9].

Nutraceuticals, which combine two words, nutrient and medicinal component (pharmaceutical) [9], simply depict food extracts/products that possess health benefits, ranging from delivery in the form of functional foods/ingredients to disease prevention/treatment [2]. Nutraceuticals, including vitamins, minerals, and essential fatty acids, from different sources have strong health improvement properties and can delay the process of aging, increase life expectancy, prevent chronic diseases, and/or improve the body function/structure [4, 10]. Currently, nutraceuticals have gained many interests because of their potent nutritional properties, therapeutic effects, and relative safety. Marine nutraceuticals comprise dietary/food supplements that contain bioactive compounds, which include oils rich in long-chain omega-3 polyunsaturated fatty acids (LC w3-PUFA), such as eicosapentaenoic acid (EPA or 20:5 w3), docosapentaenoic acid (DPA or 22:5 w3) and docosahexaenoic acid, chitin, chitosan and associated products, enzymes, peptides, and vitamins [2]. Natural nutraceuticals, like those found in seafood, are also well positioned to improve the quality of life and prevent health challenges. What makes the marine nutraceuticals desirable/safe is underpinned by their nontoxic nature [9]. Fish/marine species comprise approximately one-half of the global biodiversity—a massive resource for novel compounds [5]. The global population, however, is still confronted by various health challenges, from cardiovascular disease, diabetes, and obesity to hypertension. In fact, cardiovascular disease constitutes among the most common causes of global morbidity/mortality, exasperated by the elevation of blood lipids [5]. Reducing the low-density lipoprotein-cholesterol (LDL-C) helps in preventing cardiovascular disease, especially coronary heart disease [11]. Consumption of (cold-water) marine fish/artic mammals rich in *Ω*-3 (or n-3) polyunsaturated fatty acids (PUFAs), particularly eicosapentaenoic acid (EPA, 20:5 n-3) and docosahexaenoic acid (DHA, 22:6 n-3) can help to lower the incidence of coronary artery disease [5, 12]. As such potential benefits associated with fish consumption are reflected by bioactive and nutraceutical aspects,there are evidenced successes of biological properties as well as nutraceuticals from fish/marine sources still persist [13]. Fish-based nutrients should, therefore, be the way to go particularly from the global food security perspective [13, 14].

Moreover, research investigations involving marine-derived molecules are on the rise, with new bioactive compounds emerging with promising properties, strengthening the position of fish-based nutrients as nutraceuticals. A summary of major reviews conducted on various bioactive/nutraceutical aspects of fish/marine products is presented in Table 1. Ashraf et al. [1] reviewed fish bioactive components and their application as nutraceuticals for therapeutics in treating chronic diseases, as well as ethnic issues related to fish consumption or its by-products, and Šimat et al. [9] provided an update of functional seafood compounds (from chitin and chitosan to phenolic compounds/minerals) particularly on their potential use as nutraceuticals and health benefits; Hosseini et al. [15] reviewed the aquatic-sourced bioactive ingredients and their potential application in the food, supplement, and pharmaceutical industries, supplemented with key technofunctional and sensorial attributes plus their gastrointestinal fate/potential toxicity. Other researchers looked at nutraceutical values of fish based on ecogenomics data, limitations on climatic influences, multiple conservation constraints/implications [16], utilization of marine bioactive by-products, and potential applications in the food/pharmaceutical industries [13]. How n-3 PUFAs and bioactive peptide components from fish influence cardiovascular disease risk factors, as well as main clinical trials that either support or do not support this association [5]; marine-based nutraceuticals, from isolation, identification, and characterization of (marine-derived) bioactive compounds with their diverse therapeutic potentials [14]; the important functions and therapeutic potentials of marine fish-derived bioactive peptides/proteins for human therapy [17]; bioactive peptides derived from marine organisms and their biological activities with potential applications [18]; and marine nutraceuticals, their application, and their health benefits [2] are among the earlier reviews. The abovementioned reviews clearly show that the knowledge base of bioactive/nutraceutical aspects of fish/marine products is steadily on the rise. Therefore, there is a need for continuous synthesis of relevant literature(s) to provide increased clarity as well as enhance the understanding that challenges this specific subject area. In this current review, we highlight important information regarding bioactive compounds and therapeutics obtained from fish, specifically revisiting their suitability in functional foods to enhance human health. This contributionis hereby constructed as follows: (a) fish nutraceutical/therapeutic components, (b) constituents of fish-based nutrients and their suitability in functional foods, (c) fish antioxidant/bioactive compounds to help alleviate health conditions, (d) common human ailments alleviated by fish-based nutrients, and (e) role of fish in mental health and immune system. At the end of this work, in addition to concluding remarks, we provide the direction of future studies.

## 2. Fish Nutraceutical and Therapeutic Components: A Primer

### 2.1. Proximate and Mineral Composition of Fish and Its Oil

Fish (and fish products) is well known to offer numerous/unique nutritional health benefits. Fish as an essential human nutrient resource, therefore, requires increased global awareness.  Figure 1 shows the proximate and mineral composition data considered representative of a typical fish. Specifically, the proximate composition comprised moisture, protein, lipid, and ash content estimated from 62 species of fish as reported by the FAO [19], whereas the mineral compositions comprised sodium (Na), magnesium (Mg), zinc (Zn), potassium (K), phosphorus (P), iodine (I), calcium (Ca), iron (Fe), and selenium (Se) [20–23]. Clearly, fish possesses protein alongside several amino acids, dietary vitamins (A, B3, B6, B12, D, and E), minerals (calcium, iron, phosphorus, zinc, iodine, and selenium), PUFAs, and several other micronutrients [14, 21, 24]. Further, Figure 2 shows the composition of fish oil, from fatty acids compared to the others. Specifically, fatty acids comprised PUFA, MUFA, and SFA, whereas other compositions include sterols, vitamins, minerals, polyphenols, and pigments. Fish importantly comprise long-chain omega-3 fatty acids, EPA (eicosapentaenoic acid), and DHA (docosahexaenoic acid). DHA is crucial for brain development in children, whereas ALA (alpha linolenic acid) is a precursor of DHA [25]. Beneficial to humans, the daily intake of 250 mg EPA+DHA can prevent CHD [26] and 150 mg/day for optimal brain development. Besides the proximate composition of fish and fish-based products, the principal muscle constituent includes protein, water, and lipids, representing about 98% of the overall weight [1].

Given that fish consumption for good health steadily increases worldwide, many biotech researches strive to create new, functional food and pharmaceutical (fish-based/sourced) items. Polyunsaturated fatty acids (PUFAs) in fish oil, reflected strongly by bioactive lipids, comprise both eicosapentaenoic acid (EPA) and docosahexaenoic acid (DHA), which are largely associated with lowering the prevalence of heart disease across fish-eating communities [27, 28]. Fish oil consumption would minimize arterial stiffness and lower the incidence of heart diseases due to the presence of EPA and DHA, which help to lower blood pressure. Apart from its oil, other important elements found in fish, like proteins, fat, minerals, and vitamins, remain very helpful for human wellbeing [29, 30]. With the increasing human population and per capita income, the demand for fish and products continues to rise [25]. Besides, about 50% of fish consumed today emanates from aquaculture farms, despite the differences in nutritional composition between cultured and wild fish species. A minor difference between these two sources is the quality and quantity of fat. For instance, carps, tilapia, and clarias are among the most commonly farmed species, with long-chain omega-3 content lower than those contained in wild species, such as salmon. Nonetheless, the culture species is still a good source of omega-3 acids when compared with meat and beef sources. The merit of farmed fish includes consistent nutrient composition given the monitored feed and water quality, unlike the wild species that feed on whatever is gotten from the environment [25]. Tørris et al. [31] also stated, “In many nations' diets, fish is a great source of nutrients such as minerals, vitamins, vital fatty acids, and proteins. 80 percent (*w*/*w*) water, 8–25 percent proteins, 0.5 percent–30 percent fat, and 0.6 percent–1.5 percent mineral compounds make up the composition of fish. Water-soluble vitamins abound in fish, and fish oil (especially from the liver) is high in vitamins A and D.”

### 2.2. Further Insight into the Compositions and Nutraceuticals in Fish Products

As reported by FAO [19], fish muscles comprise mainly proteins (9–24%), water (59.1–87.8%), lipids (0.8–23.5%), and ash (1.6–6.2%), which amounts to 98% of the total body weight. When compared with meat, fish is believed to possess considerably enhanced essential amino acids together with such other nutrients like zinc; iron; vitamins A, D, E, and K; minerals; iodine; phosphorus; and micronutrients [24]. Nerhus et al. [22] reported fish mineral components such as sodium (72 mg), potassium (278 mg), phosphorus (190 mg), magnesium (38 mg), calcium (79 mg), selenium (1.2 mg), zinc (1.6 mg), iodine (0.13 mg), and iron (0.12 mg), which makes it very pertinent to human diet. The nutritive composition of fish would vary given to such factors like age, sex, temperature, and feeding habits [20]. Besides preventing or treating various diseases, the nutraceutical benefits of fish consumption remain key for human wellbeing and physiological functions [32], which some workers believe help delay the aging processes and increase life expectancy [33] (Table 1). More so, fish remains a cheap nutraceutical resource with the capacity to help solve nutritional problems especially for the most vulnerable and low-income earners [34].

Some major nutraceutical components of fish and their health merits are presented in Table 2. For example, omega-3 and omega-6 are believed to be available in spiny dogfish, mackerel, salmon, sardines, and anchovies [35, 36]. Other fish species rich in iron and zinc include Sperata seenghala and Rita rita [37]. Vitamins A and D can also be found in *Amblypharyngodon mola* [8], whereas methionine, serine, alanine, and leucine are believed to be, respectively, found in *Stolephorus waitei*, *Mugil cephalus*, *Polypedates maculatus*, and *Lethrinus harak* [38–42]. Moreover, aspartic and glutamic acid are also believed to be found in Labeo niloticus [41], whereas arginine, isoleucine, tyrosine, and proline are believed to be found in Oncorhynchus mykiss [40]. Importantly, several communities across the globe depend on these (above-named) fish species. Additionally, the regular consumption of fish, like at least 1-2 servings weekly, would provide about 200-500 mg dose of omega-3 fatty acids, which can prevent various heart diseases and stroke in humans [43], which further reiterates the therapeutic properties of fish [44]. Besides fish consumption constraints that still persist especially in the poorer communities of today's world, both food and pharmaceutical industries equally encounter challenges regarding their processing [16].

## 3. Constituents of Fish-Based Nutrient and Their Suitability in Functional Foods

### 3.1. Proteins and Its Amino Acids

Proteins remain among key macromolecules that serve as nutrients, antibodies, transport molecules, hormones, etc. In addition to their support for human growth, development, and body tissue maintenance, proteins regulate key metabolic pathways and act as precursory molecules for the synthesis of substances with biological importance [45]. More so, other benefits of proteins have been reported, for example, prevention of protein-calorie malnutrition [1]. Fish-based protein (example from sardine) would modulate several regulatory factors including lowering insulin resistance, leptin, and tumor necrosis factor- (TNF-) *α*, improving hyperglycemia, and decreasing adipose tissue oxidative stress in animal models [46]. In terms of nutrition, the human body readily digests and absorbs fish proteins, so asto deliver important biological effects [47]. Bioactive peptides (called hydrolysates) have been isolated from different species of fish [48]. Such fish protein hydrolysates, gotten via hydrolysis of protein, possess important metabolic activities, from antioxidant, antimicrobial, to antihypertensive aspects [49, 50]. The biological activities of fish muscle protein hydrolysates promise potential application to functional food/nutraceutical industries. Fish protein hydrolysates possess antiobesity, immunomodulatory, antioxidant, angiotensin I-converting enzyme- (ACE-) inhibitory, antimicrobial, and anticancer activities at in vitro models [51]. Low molecular weight fish protein hydrolysates, which largely exhibit superior bioactivities, require special attention given their safer and natural sourced contribution to disease management over synthetic drugs. The antiobesity activity is exerted via secretion of satiety hormones, stimulation of lipolysis, and inhibition of digestive enzymes and adipogenesis. Immunomodulatory activity is conferred by activation of MAPK or NF-*κ*B signaling pathway, regulation of inflammatory mediators (NO, iNOS, and COX-2), proinflammatory cytokines (IL-6, IL-1*β*, and TNF-*α*), and anti-inflammatory cytokines (IL-4, IL-10) [52–55]. The antioxidant effect is by radical-scavenging, ferric-reducing, and metal-chelating activities [51]. The ACE-inhibitory activity of hydrolysates is by effective interaction with ACE through hydrogen bonding and hydrophobic interactions with amino acids at the active site of ACE, hence reducing the catalytic activity of ACE [56, 57]. Several fish species including tuna, shellfish, salmon, sardine, and bonito have been shown to be great sources of ACE inhibition [58]. Furthermore, ACE peptides/inhibitors extracted from fish and fish products would possess antihypertensive activity, to hinder the accumulation of cholesterol plaques within the inner arterial walls and reduce blood pressure [59].

Adding as rich sources of amino acids and peptides, fish proteins remain highly digestible especially in balanced proportions. The digestibility of such components as amino acids and proteins is critical to the bioavailability and therapeutic effects of fish products [60]. Balami et al. [46] understood that about 60% of the inhabitants in developing countries depend on fish,which constituted about 30% of their animal protein supplies. Essential for the development of the human body, growth, and replacement of worn-out tissues, proteins act as immunoglobulins and help to maintain the water balance [61]. Amino acids build the protein block and sustain the metabolic pathways. Their deficiency, however, affects metabolism and homeostasis resulting in mental disorders. Another instance is gelatin, which is derived by heating collagen at a high temperature. It has a low melting point, yet colourless and tasteless, with pharmaceutical applications especially vitamin microencapsulation [62]. Gelatin extracted from warm water fish resembles those from mammals [63]. Another typical example is collagen, which contains glycine, proline, and hydroxyproline and can be converted to gelatin when heated. Classified as the main structural protein and important in the formation of tissues, organs, and expression of cells, collagen can help in treating hypertension, as a hemostat, skin substitutes, drug delivery, and cell human implants [64]. Biologically and nutritionally required, fish proteins serve an important role in food systems, including as hormones, transport proteins, and antibodies, while the body digests and quickly absorbs them [47, 65, 66]. Bioactive peptides can be produced through protein hydrolysis especially those isolated from several fish species. They can be transported via the intestinal enterocytes before reaching circulation, where they exert favorable biological actions. Peptides can deliver a variety of biotechnological products with improved bioactive qualities, with antibacterial, antioxidative, and antihypertensive properties [67]. Antioxidant activity of fish protein hydrolysates (FPH) is strong, including the FPH hydrolyzed from tuna, mackerel, and other fish species. Lysine and methionine are two of the essential amino acids found in considerable amounts in fish protein [66]. Angiotensin I-converting enzyme (ACE) is inhibitory peptides from fish sources originally present in sardine flesh [68]. ACE inhibitory peptides have now been found in a variety of fish species, including shellfish, tuna, bonito, salmon, and sardine. Crude fish protein hydrolysates containing ACE inhibitory peptides can also be derived from refined catfish protein hydrolysis. Soluble protein fraction includes the majority of the ACE inhibitory peptides [68]. Among the water-soluble protein components, glutamic acid, proline, taurine, glycine, and alanine are abundant in fish muscles. Taurine is also a very necessary amino acid linked to some aspects of mammalian development and is abundant in fish and able to lower blood pressure, enhance heart function, and lower cholesterol levels. Cod, mackerel, salmon, albacore tuna, ray, shark, and numerous other species contain taurine, for instance, white fish that contain more taurine than fatty fish [7, 69]. Most effective free amino acids that interact with free radicals are those that can easily give away hydrogen atoms, such as cysteine and methionine, which have nucleophilic sulfur-containing side chains or aromatic side chains: tryptophan, tyrosine, and phenylalanine. Cysteine, methionine, lysine, taurine, tryptophan, tyrosine, and phenylalanine are the particular molecules, which are responsible for the bioactivity of fish hydrolysates. Antihypertensive peptides (ACE inhibitors) found in fish and fish extracts can help to reduce blood pressure and prevent the deposit of plaque of cholesterol on the inner walls of arteries, the latter activity specifically believed to impede the blood flow [70]. A sulfonic acid group, not integrated into proteins, is the one having abundant free amino acids in tissues, including skeletal, brain, and cardiac muscles [71].

As unitary components of protein, amino acids are very important for various physiologic and therapeutic functions in the body. As per the report of Kundam et al. [58], fish muscles contain several amino acids majorly glutamate, glycine, taurine, arginine, proline, and alanine, while the essential amino acids predominant in fish proteins are lysine and methionine [47]. The aromatic (tryptophan, tyrosine, and phenylalanine) and nucleophilic amino acids containing sulfur side chains (cysteine and methionine) are more efficient in terms of bioactivity of fish hydrolysates because of their ability to easily give away hydrogen atoms and interact with free radicals [58]. The most remarkable bioactivities of fish-based hydrolysates are dependent on their amino acid composition and structural and conformational characteristics [51]. Of special interest is the conditionally essential amino acid called taurine. Taurine has been found abundantly in several types of fish including wild salmon, mackerel, cod, tuna, albacore, shark, and ray and has been shown to be involved in some aspects of mammalian development [58]. Taurine contains a sulfonic acid group instead of the usual carboxylic acid moiety in amino acids. The potentiality of taurine has been tailored towards its usage as a therapeutic agent against congestive heart failure and several other disease circumstances, including reduction of blood pressure, improvement of cardiac performance, and reduction of blood cholesterol levels [72, 73]. Taurine possesses cytoprotective activity, which it exerts via major mechanisms including antioxidation, energy metabolism models, gene expression, modulation of endoplasmic reticulum stress, neuromodulation, quality control, Ca^2+^ homeostasis, and osmoregulation [73–82].

### 3.2. Essential Fatty Acids

Fishes contain polyunsaturated fatty acids (PUFAs) and considerable levels of monounsaturated fatty acids. These fatty acids are regarded as beneficial if they are not oxidized [83]. Fish oil basically comprises two types of polyunsaturated fatty acids (PUFAs), namely, docosahexaenoic acid (DHA) and eicosapentaenoic acid (EPA), known as omega-3 fatty acids, which are readily digestible for energy metabolism and several biological activities, including protection against chronic diseases [58]. Alpha-linolenic acid (ALA) is another vital omega-3 fatty acid which is precursory to EPA and DHA. Fish consumption helps to elevate EPA and DHA in blood, consequently lowering the development of coronary heart diseases via diverse mechanisms. Fatty acids found in fish oils help protect against coronary heart disease by decreasing serum triglyceride concentration, improving cardiac function, and reducing blood pressure and inflammatory responses [59, 84]. The anti-inflammatory property of EPA and DHA occurs via modulation of prostaglandin synthesis [61, 85]. Fatty acids reduce the amount of platelet build-up in the blood, thus narrowing the blood and reducing the propensity of blood clot formations [58]. Lipid fractions of fishes are great sources of these PUFAs, which are essential for promoting human health, because humans cannot synthesize PUFAs longer than 18-carbon atoms except from diets [86]. Omega-3 fatty acids abundant in brown flesh of oily fish are very useful, in terms of conferring prevention of cardiovascular diseases [50]. Fatty fishes containing omega-3 fatty acids include mackerel, salmon, herring and sardine, eel, trout, and anchovies [87]. Omega-3 fatty acids in fatty fish are vital for the growth of children. Particularly, DHA is essential for optimal brain and neurodevelopment in children, whereas EPA is essential for the improvement of the overall cardiovascular health. Fatty acids are involved in osmoregulation, nutrient assimilation, and nutrient transport [27, 28, 46, 60]. Average daily consumption of 250 mg of EPA/DHA is recommended by the U.S. of Agriculture and of Health and Human Services [88]. Sterol molecules in lipids derived from marine sources can lower the amount of low-density lipoprotein (LDL) cholesterol in vivo. Phytosterols are also significant precursors of a number of vitamins. Gallego et al. [89] reported that “ergosterol is a precursor of vitamin D2 and cortisone.”

A 2020 data survey showed that the intake of probiotics, fish oils, vitamin D, or its combination provided a slightly lower risk of SARS-CoV-2. Although not conclusive, supplements should not be taken in place of drugs or vaccination. Elsewhere, postpartum depression in pregnant women or breastfeeding mothers could happen due to low levels of omega-3 [31, 58, 90, 91]. Fish consumption especially those rich in oils should be encouraged, although the intake requires great caution to avoid fish harbouring heavy metals. Essentially, three major types of fatty acids exist, largely classified by length, presence, and arrangement of double bonds, which include saturated (SFAs), monosaturated (MUFAs), and polyunsaturated (PUFAs) fatty acids. Specifically, the essential fatty acids function in brain development, healthy cell membranes, regulation of blood pressure and viscosity, immune responses, and production of hormones necessary for the body [31, 58, 90, 91]. Based on the position of double bonds therein, the PUFAs are largely classified into two, namely, omega-3 and omega-6. Both are able to relieve cardiovascular diseases given their varied biological roles [85]. Contributing to children growth and brain development, the omega-3 fatty acids help to prevent asthma (in children), hypertension (in adults), neurological formations, etc. [92].

### 3.3. Vitamins

Vitamins produce a wide range ofbiological effects considered necessary for many chemical and physiological processes in the human body. Fish and fish-based products are great sources of vitamins needed for the normal human bodyfunction. For instance, vitamins A, B, D, and E are understood to be widely available in fish [46, 58]. Specifically, vitamins A, D, and E are readily bioavailable in fish oils like cod liver oil and in (fish) species like sardine, mackerel, herring, lake trout, and salmon [58]. Vitamin A sustains normal growth, builds cells, and promotes good eyesight [93], yet dependent on the form in which they exist. Retinol, for instance, is converted in the body to 11-trans-retinal via an oxidative process, whereas the 11-trans-retinal is subsequently isomerized into 11-cis-retinal, which is the functional form of the vitamin essential for vision/visual physiology [94]. Additionally, vitamin A can influence the biosynthesis of many proteins that regulate the cell development/function or determine cell sensitivity to hormones and hormone-like factors and impact the formation of hormones. Vitamin D in fishes that exists in the form of cholecalciferol (vitamin D3) can abate vitamin D deficiency-related conditions, including rickets, osteomalacia, and osteoporosis [1, 95]. A link has also been established between vitamin D deficiency and diabetes, amplified proliferation of cancer cells, and increased incidence of autoimmune and cardiovascular diseases [50]. Hence, dietary vitamin D obtained from fish and fish-based products could attenuate the highlighted conditions in humans, since fatty fish is one of the very few dietary sources of vitamin D [96].

### 3.4. Minerals, Carotenoids, Chitin, and Chitosan

The great amounts of essential minerals and trace elements found in fish have been attributed to the capability of fishes to obtain inorganic atoms from aquatic bodies, thus explaining why these essential minerals are more abundant in aquatic foods than in terrestrial foods. When compared to terrestrial diets, these critical elements are found in greater concentrations in seafood [58]. Present in fish and other aquatic foods, some essential minerals like calcium, potassium, iron, sodium, iodine, selenium, magnesium, and zinc provide numerous health benefits, including important biochemical responses [1, 97]. Fish is among the most vital sources of calcium (especially fishbone) and involves in bone formation and calcified dental tissues in children, elderly persons, and pregnant women [59, 97–99]. In addition, magnesium and phosphorus are also essential in teeth and bone formation, whereas sodium and potassium help in nerve impulse transmission and electrolyte balance maintenance. Iron is a component of hemoglobin that transports oxygen around the body [100, 101]. Zinc acts as a cofactor in the activity of over 300 enzymes that are essential for metabolism, DNA and protein synthesis, digestion, nerve function, development and function of immune cells, cell growth, and division [102–105]. Saltwater fish and other sea foods are natural sources of dietary iodine; the latter is essential in making thyroid hormones that control human growth and development. When deficient, lack of iodine can cause intellectual disability, cretinism, and other additional risks especially in pregnancy [106]. Besides the formation of bone and teeth, other minerals like potassium, magnesium, sulfur, zinc, copper, and iodine commonly found in the flesh of fish deliver electrolyte balance and bone formation and serve as a cofactor of enzymatic reactions and hemoglobin molecules [46, 101, 107].

Carotenoids can occur in various forms in fish.Typical examples include beta carotene (orange in colour), lutein (greenish-yellow), alpha- and beta-doradexthins (yellow), canthaxanthin (orange-red), and astaxanthin (yellow in colour), which as pigments are responsible for giving fish a wide range of colour. The most common appears to be astaxanthin, which is able to prevent eye macula (lutein and zeaxanthin) that comes from damaging blue lights and oxidative stress [108]. Chitin and chitosan are extracted from shells of marine crabs and shrimps as it is a major component of their exoskeleton. They also help in structural support and protection [109]. Also, as a structural polysaccharide, chitosan is less expensive, as it is obtained when the acetyl group derivatives are removed from chitin polymers. Both chitin and chitosan provide health benefits such as wound healing, immune system stimulant, antiulcer agents, bactericide, antioxidant agent, and antiaging cosmetics [110, 111]. Also, chitin/chitosan is useful for nutraceutical applications and can be augmented by stimulating the assimilation of derivatives like fibers, film, and chitosan-based nanomaterials, being commercially available nontoxic/natural substances [60, 112–114]. In general, chitosan has found wide applications in nanoencapsulation of many nutrients and bioactive compounds found in foods, including fish, where it helps in nutrient delivery, absorption, and protection [60, 112, 115, 116]. It has wide use in many pharmaceutical, nutrition, and biomedical applications [112–114].

### 3.5. Farmed Fish vs. Wild Fish

The nutritional and bioactive compositions of both wild and farmed fishes vary. In wild fish alone, for instance, the levels of nutrients and bioactive compounds can significantly vary even within the same species. Nutrients in farmed fishes, especially fatty acids, are usually influenced by feed consumption. Farmed fish contains higher or similar total amounts of long-chain omega-3 PUFA and also higher fats than wild fish [117, 118]. When raised under suitable conditions, nutrients and bioactive compounds in farmed fish are considered beneficial as those in wild fish, including for preventing diseases, such as cardiovascular diseases, with the advantages of being fresh and apparently not toxic. However, there are likely to be some differences in levels of certain nutrients and bioactive compounds. For example, wild salmon usually have lesser calories, vitamins A and D, and saturated fat than farmed salmon; however, it has more protein content [119]. In both farmed and wild salmon, omega-3 fatty acids often vary based on the salmon's feed. Sprague et al. [120] reported slight variations in iodine content of farmed and wild fishes. Consumers have different perceptions about farmed and wild fishes. In general, fish consumers believe that there are considerable differences between farmed and wild fishes, with many having preferences for wild fishes, although the consumption of farmed fishes has been growing remarkably worldwide [121].

## 4. Fish Antioxidant/Bioactive Compounds to Help Alleviate Health Conditions

Nutrients in food, at their most basic level, nourish and promote the ability of our body to stay fit. However, due to additional health benefits from food, such as the prevention or treatment of specific diseases, white fish, for example, cod, hake, and plaice, contains almost 20% protein, 80% water, and 0.5-3% oil, with minimal vitamins, minerals, carbohydrate, and other nutrients [31]. Similarly, fatty fish have around 20% protein, but their water (62-70%) and oil levels are much higher (10-18%). During digestion, the protein in oily and white fish is broken down into polypeptides, amino acids, and peptides. Because the majority of them contain bioactive qualities, they are called bioactive chemicals. Bioactive chemicals are additional nutritional ingredients found in meals that are naturally present in small amounts. These compounds have been shown to be helpful to human health [69, 122, 123]. Various physiological mechanisms contribute to these health benefits, including antioxidant activity, hormone treatment, and immune system enhancement, and improve digestive tract functions, butyric acid production in the colon, and absorption and dilution of substances in the gut. Food-related diseases such as cancer, diabetes, hypertension, and obesity have encouraged individuals to seek out meals and food items that give both functional and health advantages. Peptides and other antioxidants have shown antihypertensive properties in vivo, and different other studies show bioactivities as well as antiproliferative and antibacterial activities in vitro [124].

Table 3 shows the therapeutic functions of fish-based nutrients and bioactive compounds in several diseases. Disease conditions outlined in this context include diabetes, cancer, cardiovascular diseases, obesity, brain function/immune system disorders, and oxidative stress-related diseases [58, 96, 125–129]. Clearly, there is a wide range of bioactive compounds associated with fish species, which provide an array of nutritional benefits/therapeutic effects.  Table 4 shows fish by-products as an important source of nutraceuticals and functional foods. The fish by-products provided in this context include scales, skin, bones, ground skin, head, belly part, trimmed muscle, frame, entrails, head and backbone, gill and intestine, and cartilage [130–141]—all of which provide varied functional products, nutritional purposes, and pharmacological activities. The therapeutic functions of fish-based nutrients and their bioactive compounds tend to draw a great deal of attention. As substances that can inhibit oxidation by free radicals in the body, even at low quantities, antioxidants generally work to defend our bodies from oxidative stress as well as disease progression [142]. Antioxidant properties of a chemical are demonstrated by its ability to treat degenerative illnesses like cardiovascular disorders, cancer, inflammatory disorders, and diabetes [123].

The reactive oxygen and nitrogen species (ROS and RNS) are created spontaneously in cellular metabolism. However, RNS and ROS assault the cell membranes in the body, resulting in numerous fatal illnesses if not reversed. As a result, the body manufactures its own endogenous antioxidants to combat the ROS and RNS' actions [27]. Antioxidant properties have been demonstrated in fish protein hydrolysates from tuna and mackerel [124]. The antioxidant properties of peptides and hydrolysates of fish are beneficial to one's health, as evidenced by antioxidants' ability to defend the body against RNS and ROS molecules, which attack the protein, membrane lipids, and DNA, resulting in degenerative diseases such as cardiovascular disorders, dementia, diabetes, obesity, and cancer [159]. Fish peptides/hydrolysates have antioxidant capabilities such as scavenging ROS free radicals and preventing oxidation of cell membranes, which is ROS-induced. The efficacy of fish protein hydrolysates or peptides is determined by the size of peptide and amino acid composition [160]. To avoid the possible hazards posed by synthetic antioxidants, antioxidants acquired through dietary sources have recently become popular. Fish have antioxidant potential, especially in vitro antioxidant activity demonstrated in peptides from mackerel or fish protein hydrolysates [7]. Peptides extracted by the hydrolysis of mackerel fish muscles would utilize protease N inhibiting autoxidation of linoleic acid. Protein hydrolysates of tilapia fish could have antioxidant properties. With an elevation in the rate of hydrolysis of salmon fish muscle, lower molecular weight peptides and hydrolysates have been identified, which boost the free radical scavenging capability of the salmon fish muscle hydrolysate [161]. Tuna fish protein hydrolysate can inhibit the hydroxyl radical-induced damage in DNA, which demonstrates the antioxidant activity. DNA damage would bring about an onset of various grave diseases, including coronary heart disease, diabetes, and cancer [27]. As a result, frequent fish consumption might help to prevent or treat such illnesses.

## 5. Common Human Ailments Alleviated by Fish-Based Nutrients

### 5.1. Cardiovascular Disease (CD)

The bioactive compounds in fish play a very critical role in the management and prevention of wide range of specific health conditions. For instance,on one hand, there is a link between high triglyceride levels and high blood clotting factors in diabetics and overweight people. Naturally, such type of interaction may increase the chances of blood clotting and severely damage the normal activity of the cardiovascular system. Intake of fish oil, on the other hand, can help reduce the level of triglycerides in the blood, thereby limiting the chance of blood clots in the circulatory system and this has been supported byepidemiological studies [31].

Aluko and Aluko [96] has been quoted to emphasize that“when two fish dinners (300 g) per week were incorporated into the diet of individuals suffering from myocardial infarction over a two-year period, there was a 29% reduction in all-cause death; this link was much greater in diabetic women, with a 60% decreased incidence of coronary heart disease (CHD) in the group with the greatest fish intake when compared to those that ate little or no fish; even in individuals who had already established CHD, just 150 grams of fish per day reduced the chance of major health consequences.” From this quote, the authors believe that the presence of omega-3 PUFAs in fish is largely associated withcardiovascular health benefits. There is evidence that omega-3 PUFAs to the diets of CD patients was associated with a significant reduction in cardiovascular fatalities and their associated symptoms. More so, the levels of omega-3 fatty acids in the blood are inversely corrected with the risk of cardiovascular diseases, including stroke and sudden death from CD [12, 91]. Thus, the reduction of triglyceride and cholesterol levels in blood serum after taking fish oil demonstrates this. Whereas the consumption of saturated fatty acids raises blood pressure, an increase infish consumption would largely raise the blood levels of DHA and EPA, which would help to decrease the blood pressure. From this, there is a strong link between eating fish and lowering CVD and CHD, which is opined to exemplify the beneficial effects. More so, those who consume predominantly marine foods, such as Alaskans and Japanese, have less cardiac problems [91].

The delivery of health benefits by fish consumption includes lowering the risk of ventricular fibrillation, commonly seen after myocardial infarction. Fish oil in the diet of hypercholesterolemic animals would decrease the risk of atherosclerosis and arterial stiffness. Aluko and Aluko [96] also reported that “dietary fish oil raised the content of long-chain and n-3 polyunsaturated fatty acids (PUFA) in cardiac cells as compared to the control in a rat model of myocardial dysfunction.” Based on this premise, the authors herein concur that fish oil intake may well help to reduce platelet clumping in the circulatory system. Fish oil treatment would lower pathological alterations associated with ischemia-reperfusion, such as decreased cardiac contraction force, increased coronary perfusion pressure, and ventricular arrhythmias. Fish oil consumption, therefore, would positively enhance the heart, considering the omega-3 fatty acids as among the key bioactive components. Given by cis-isomer as the most bioactive form, the beneficial health effects of PUFAs would be reflected by their isomer structure [96]. Cis-configured fatty acids have a stiff nonlinear structure that improves membrane fluidity when introduced into cells. Increased fluidity of the membrane improves cell-cell communication and aids either the maintenance of normal homeostasis or the prevention of metabolic diseases [96].

### 5.2. Cancer

Cancer is a medical condition in which cells continue to grow and divide in an abnormal fashion. By attacking and destabilizing the regular biological tissues, these cells could result in the eventual death of humans if not tackled. On this basis, the promotion of apoptosis continues to be a major target for anticancer treatment [162]. The relationship between cancer inhibition and fish consumption has been studied extensively. Kim and Wijesekara [145] investigated fish protein hydrolysates' antiproliferative effectiveness in breast cancer cells. The hydrolysates were found to include a multifarious combination of free amino acids and peptides with varying molecular weights ranging up to 7 kDa, as well as lower amounts of lipids and sodium chloride. Omega-3 fatty acids were tested in animal studies for their antitumoral and antimetastasis properties. Ulagesan et al. [163] claimed that “the mice were provided an omega-3 fatty acid-rich diet and a number of characteristics were monitored, including tumor development, body weight, and lung metastasis. Soybean oil was included in the control diets. These diets were put to the test in conjunction with the cytotoxic drug cisplatin. Fish oil inhibited tumor development and decreased the number of metastatic sites.” Despite the paucity of evidence on the beneficial benefits of fish-eating on the formation and progression of cancer, research suggests that fish ingredients may provide some protection against tumor growth [164]. Particularly, foods containing omega-3 polyunsaturated fatty acids such as DHA and EPA, especially those high in omega-3 polyunsaturated fatty acids, as EPA and DHA, are believed to help prevent tumor growth. In those with familial adenomatous polyposis, EPA in the diet is believed to lower the number and size of rectal polyps (FAP). Moreover, fermentable fiber in the diet can significantly boost the anticancer properties of fish oil, given by the creation of butyrate from fiber fermentation, which works in tandem with the fish oil PUFAs (notably DHA) to destroy cancer cells. More so, the fish oils and vitamin D help colon epithelial cells develop more successfully, to minimize the likelihood of genetic alterations that lead to new unwanted characteristics [164].

### 5.3. Diabetes and Obesity

In animal studies, insulin resistance was lowered by fat-free fish protein diets, indicating that such diets could be beneficial in human glucose regulation. Animal research was done and showed that cod protein is useful in a high-fat, high-sugar diet. Insulin sensitivity studies showed that the quantity of glucose required to induce hyperglycemia in cod-fed rats was much larger than that in casein-fed rats, indicating that it protected rats from developing obesity-related insulin resistance and glucose tolerance. In comparison to casein, cod protein increased insulin-dependent glucose absorption, implying greater insulin sensitivity. Insulin sensitivity was found to be connected to a reduction in fat deposition and weight gain. Humans were fed cod protein, which showed a similar result [159]. Other workers like Tufail et al. [165] considered obesity as a metabolic condition emerging from energy intake that exceeds the energy expenditure. In fact, both Tufail et al. [165] and Yasmin et al. [166] considered the pathophysiology and etiology of obesity and diabetes mellitus as crucial conditions that pose a significant threat and economic burden to humans, globally. Increasingly becoming a major medical problem worldwide, obesity projects a negative societal impact on human girth [166]. Clinically, fish oil can help people lose weight. Thus, through fish consumption as compared to meat, the body mass index (BMI) can be lowered. It is believed that by blocking important enzymes responsible for lipid syntheses, both DHA and EPA would help reduce obesity and prevent the entry of free fatty acids into adipocytes for lipogenesis [71]. When compared to casein, salmon diets help to reduce weight of epididymal white adipose tissue caused by dietary fat [96].

Increased deposits of the white adipose tissues, which are connected to insulin resistance and increased water retention, are a warning sign of the start of obesity. These findings show that not only does eating fish protein enhance energy expenditure but it also improves insulin sensitivity, decreases water retention in the body, and, as a result, reduces body weight, hence regulating obesity [71]. Protein diets, among other things, have a satiating effect, which supports the weight reduction seen with increased fish consumption. Because the satiating effect reduces food intake and overall calorie intake, instead of fat being stored in adipose tissue, leading to weight increase, the proteins are integrated into the lean muscles [71]. Functional foods/meals having fish-based nutrients can help weight loss to be achieved in a practical and beneficial way, which would decrease cholesterol, increase satiety, as well as increase fat oxidation rates. Also, functional foods/meals can help to reduce the total adipose tissue to actualise a healthy body weight. Functional foods, when combined with a healthy diet and regular exercise, can significantly help with weight reduction and control [129].

## 6. Role of Fish in Mental Health and Immune System

Fish consumption benefits the human brain in several ways, including depression reduction, early-stage growth, and the nurturing and maintenance of cognitive activities in older years of life. Omega-3 fatty acids, i.e., PUFAs, contained in fish oil, as well as in various natural antioxidant components that generally stop oxidative degradation of the PUFA omega-3 fatty acids in the fish, provide these beneficial effects. Regular dietary fish consumption has been shown to reduce depressive symptoms in individuals [71] elderly. The massive quantity of DHA pumped into the retina and brain underpins a good relationship between fish consumption and foetal development and early life. Because of the structural frame of the cis-double bonds, solid linear packing of DHA is not feasible; therefore, high amounts of this fatty acid result in increased cell membrane fluidity in the retina and brain. As a result, the DHA-engineered fluid cellular structure is believed to improve organ performance via enhanced competence of signaling mediators—a few of which, like ions, eicosanoids, and sugars, are required to flow in and out of cells. Some workers showed that prematured neonates were provided DHA-enriched meals, their brain and retina performance improved, but those who were not fed DHA lacked normal cognitive and retina functioning. In addition, kids born to mothers who ate fish oil-rich diets during their pregnancy grew up to possess a higher cerebral and problem-solving capability, together with superior hand and eye motions. More so, fish oil has been shown to reduce the cognitive decline in the elderly [27]. Besides being associated with reproductive health, fish oil consumption remainsessential for healthy eyesight and brain development, gievn the function that DHA serves to the brain nerves. Holistically, omega-3 fatty acids present in fish oil is crucial in the body growth and development especially to improve the reproductive system, brain, and other organs [71].

When the immune cells of the body collect DHA and EPA, the risk of inflammation is dramatically reduced. EPA and DHA replace proinflammatory fatty acids such as arachidonic acid and omega-6 PUFAs with frequent dietary fish oil consumption (anti-inflammatory fatty acids). Aluko and Aluko [96] has been quoted with the following: “consumption of 150 g of salmon three times a week resulted in lower levels of proinflammatory indicators such as C-reactive protein, interleukin-6, and prostaglandins, indicating improved immune function.” Besides, food intolerance is less common among pregnant women who consume a lot of fatty fish, and their children are less likely to have respiratory problems. Fish consumption throughout childhood is not linked to an increased risk of asthma development. Adults who consume insufficient amounts of fish in their diet are more prone to develop asthma or allergies [27]. The system of the digestive tract in ingestion of fish oil, like the immune system, has several assistances in the prevention of a variety of digestive tract problems, such as inflammatory bowel disorders. Moreover, elevated fish oil consumption would enhance the accumulation of DHA and EPA to replace PUFA n-6 (arachidonic and linoleic acids) in cell membrane phospholipids, which facilitates the beneficial/functional effects on the (cell membrane) receptors. Additionally, increasing fish oil consumption generally results in a rise in butyrate levels in the gut. As a consequence, your bowels will be healthier.

## 7. Concluding Remarks and Future Outlooks

The enormous nutritional and therapeutic benefits of fish-based nutrients and bioactive compounds cannot be overemphasised. These benefits are a result of the quality of digestible proteins, minerals, vitamins, polyunsaturated fatty acids, amino acids, and other compounds which confer nutritional importance and therapeutic effects against chronic diseases like diabetes, obesity, cancer, cardiovascular diseases, brain function and immune system disorders, and inflammatory and oxidative stress-related ailments. Hence, these benefits have prompted several researchers towards harnessing these potentials in terms of incorporation and formulation of functional foods and nutraceuticals. Increased consumption of fish should be encouraged across communities, especially those in the developing world because these are where the issue of food security among their populace appears to be more of greater concern. There is also the need for an increased campaign towards harnessing the potentials of the quality proteins, omega-3 fatty acids, and other compounds that are inherent in fish and fish-based food products. The consumer/stakeholder participation in fisheries and aquaculture sector, therefore, should be intensified in order to meet the dietary fish demands of the ever-growing population. In addition, the therapeutic potentials should be exploited especially in the area of converting fish and fish-based products into functional foods and nutraceutical, which will help in tackling the issues of nutrition-related and other diseases and ultimately improving life and wellbeing of the populace.

## Figures and Tables

**Figure 1:** Proximate and mineral composition data considered representative of a typical fish.

**Figure 2:** Composition of fish oil, from fatty acids compared to the others.Specifically, fatty acids comprised PUFA, MUFA, and SFA, whereas other compositions include sterols, vitamins, minerals, polyphenols, and pigments. PUFA: polyunsaturated fatty acid; MUFA: monounsaturated fatty acid; SFA: saturated fatty acid (SFA).

**Table 1:** Summary of major reviews conducted on various bioactive/nutraceutical aspects of fish/marine products.

Objectives of literature review	Key sections	References
This review focused on fish bioactive components, their application as nutraceuticals for therapeutics in treating chronic diseases, and ethnic issues related to fish consumption or its by-products, with more emphasis on fish waste utilization	Nutritional profile of fish; fish as nutraceuticals; background of fish bioactive compounds and fishery by-products; global fish consumption and its nutraceutical market: current scenario and future trends; importance and necessity of fish bioactive components as dietary intake; challenges and complications; future perspectives and conclusions	[1]
This review provides an update on functional seafood compounds (chitin and chitosan, pigments from algae, fish lipids and omega-3 fatty acids, essential amino acids and bioactive proteins/peptides, polysaccharides, phenolic compounds, and minerals) particularly their potential use as nutraceuticals and health benefits	Marine-based beneficial molecules; health benefit of nano-based materials for bioactive compounds from marine-based sources	[9]
This review focused on aquatic-sourced bioactive ingredients and their potential application in the food, supplement, and pharmaceutical industries, adding key technofunctional and sensorial attributes as well as their gastrointestinal fate and potential toxicity	Biofunctional ingredients of marine origin; miscellaneous bioactive compounds from marine organisms; technofunctional and sensorial attributes of fortified foods with marine bioactives; gastrointestinal digestion stability of marine-derived bioactives; safety aspects of marine-derived bioactive compounds; conclusion and future perspectives	[15]
This is a short review of nutraceutical values of fish based on ecogenomics data, their handling, and limitations on climatic influences, despite the multiple conservation constraints/implications	Background; literature collection on fish ecogenomics and conservation; nutraceutical importance of fish; literature on fish ecogenomics in PubMed; issues with ecogenomics studies and their handling	[16]
This review focused on the utilization of marine bioactive by-products, as well as how their potential can be applied to the food and pharmaceutical industries	The bioactive potential of fish frame protein; functional properties of fish skin; biomedical and food applications of fishbone; the bioactive potential of fish internal organs	[13]
This review focused on n-3 PUFAs and bioactive peptide effects on cardiovascular disease risk factors, as well as main clinical trials that either support or do not support this association	n-3 PUFAs and cardiovascular risk factors; clinical trials with n-3 PUFAs: past and future; fish proteins and cardiovascular risk factors	[5]
This review summarized the widely available marine-based nutraceuticals and researches that involved isolation, identification, and characterization of marine-derived bioactive compounds with their diverse therapeutic potentials	Nutraceuticals in the global market; marine sources of bioactive molecules; marine-derived bioactive components	[14]
This review paper highlighted the important functions and therapeutic potentials of marine fish-derived bioactive peptides and proteins for human therapy	Fish protein resources; fish protein in healthcare; development of bioactive peptides from fish proteins	[17]
This was an overview of bioactive peptides derived from marine organisms and their biological activities with potential applications in different areas	Development of marine bioactive peptides; biological activities of marine bioactive peptides	[18]
This review discussed marine nutraceuticals, their application, and their health benefits	Marine lipids; food application of marine nutraceuticals; regulatory aspects of marine nutraceuticals	[2]

**Table 2:** Some major nutraceutical components of fish and their health importance.

Nutraceutical compound	Fish species rich in the compound	Health importance	References
Omega-3	Spiny dogfish, mackerel, salmon, sardines	It improves insulin sensitivity, anti-inflammatory and cardioprotective effects, and prevention of various cancers	[35]
Omega-6	Sardine, anchovies	Reduce diseases such as arthritis, hypertension, platelet aggregation, and cardiovascular problems	[35, 36]
Iron and zinc	Sperata seenghala, Rita rita	Growth and development of immune system, wound healing, breakdown of carbohydrate	[37]
Vitamin A	Amblypharyngodon mola	For bone growth and correction of poor eyesight and promotes growth	[8]
Vitamin D	Amblypharyngodon mola	Improves density of bone and avoids rickets	[8]
Arginine, isoleucine, tyrosine, proline	Oncorhynchus mykiss	Muscle formation, detoxification of ammonia, precursor to enzymatic reactions	[40]
Aspartic and glutamic acid	Labeo niloticus	For immune functions and reduction of chronic fatigue and flavour enhancer	[41]
Methionine	Stolephorus waitei	Constituent of protein, for cellular metabolism	[39]
Serine	Mugil cephalus	Homeostasis of the cells	[41, 42]
Alanine	Polypedates maculates	For biosynthesis of proteins	[40]
Leucine	Lethrinus harak	Provides energy for protein synthesis	[38]

**Table 3:** Therapeutic functions of fish-based nutrients and bioactive compounds against several diseases.

Disease	Nutrient(s)/bioactive compound(s)	Fish species/sources	Nutritional benefits/therapeutic effects	References
Diabetes	Glycine, valine, fat-free fish protein, cod protein	Nemipterus japonicus, Cirrhinus mrigala, Catla catla, Labeo rohita	Glucose homeostasis, lowered insulin resistance, glucose tolerance, improved insulin-dependent glucose uptake, and increased insulin sensitivity	[96, 125, 143, 144]
Cancer	Squalene, omega-3 fatty acids (EPA, DHA), fish protein hydrolysates, chitin	Scardinius erythrophthalmus, Tinca tinca, sharks (shark liver oil)	Antitumor and anticancer effects against ovarian, breast, lung, and colon cancers	[126, 127, 145, 146]
Cardiovascular diseases	Omega-3 fatty acids (EPA and DHA), fish oils, carotenoids	Mackerel, herring, salmon, sardines, and tuna	Lowers triglycerides and cholesterol levels in the blood, prevents arterial blood clotting and lowers blood pressure, and reduces platelet aggregation in the blood circulatory system	[58, 95, 96, 147, 148]
Obesity	PUFAs (DHA and EPA), fish protein	Salmon, Tapra fish (Opisthopterus tardoore) oil, Greenland turbot, sardines, tuna, etc.	Inhibit key enzymes responsible for lipid syntheses, like fatty acid synthase and stearoyl-CoA desaturase-1, lower lipid synthesis, inhibit lipogenesis, enhance lipid oxidation and thermogenesis, and improve satiety	[95, 96, 128, 149]
Brain function disorders	Omega-3 fatty acids of fish oil (DHA), fish muscle protein, collagen, gelatin, fish oil, fish bone, etc.	Fatty fishes (salmon, tuna, herring, trout, sardines, albacore, etc.)	Depression-lowering effect, improve cognitive, reproductive, and retina functions and intrinsic antioxidant effects, enhance foetal development, and mitigate intellectual deterioration	[58, 84, 96]
Immune system disorder	Fatty fish oil, omega-3 fatty acids, melatonin, taurine, tryptophan, polyamines, etc.	Salmon, tilefish, tuna, trout, herring, mackerel, sardines, pollock, albacore, halibut, etc.	Immunoregulatory effect; improve immune function by reducing levels of proinflammatory markers, reduce food intolerance, and reduce risk of asthma development	[58, 96]
Oxidative stress-related diseases	Fish protein hydrolysates, protease, fish muscle protein, bioactive peptides	Tuna, mackerel, yellowfin sole, Alaska, pollock, tilapia, salmon	Antioxidant effects, prevent hydroxyl radical-induced DNA damage	[68, 145]

**Table 4:** Fish by-products as important source of nutraceuticals and functional foods.

By-product	Fish species	Functional product	Type of nutrient involved	Pharmacological activity	References
Scales	Lutjanus sp.	Chitin and chitosan	Polysaccharide-based secondary metabolites	Antioxidant, antimicrobial, antiviral, and antihypertension	[130, 133]
Skin, bones, and scales	Epinephelus sexfasciatu, Lutjanus argentimaculatus, Rastrelliger kanagurta, Pristipomoides typus, Thunnus albacares	Gelatin	Protein-based secondary metabolites	Antioxidant activity	[130, 150, 151]
Ground skin	Rastrelliger kanagurta	EPA and DHA	Lipid-derived secondary metabolites	Anti-inflammatory, antihypertensive, antidiabetic	[130, 152]
Head	Thunnus tonggol, Echinorhinus brucus	DHA, omega-3 and omega-6 fatty acids	Lipid-derived secondary metabolites	Anti-inflammatory, antihypertensive, antidiabetic	[130, 138, 139]
Belly part, trimmed muscle, frame bone, and skin	Salmo salar	Oil	Lipid-based secondary metabolites	Free radical scavenging activity	[130, 153]
Skin	Gadus macrocephalus	Gelatin	Protein-based secondary metabolites	Antioxidant activity	[154]
Skin	Johnius belengerii	Peptide	Protein-based secondary metabolites	Antioxidant activity	[155]
Skin	Rachycentron canadum	Gelatin derivate	Protein-based secondary metabolites	Antioxidant activity	[156]
Entrails, head, and backbones	Gadus morhua	Hydrolyzed proteins	Protein-derived secondary metabolites	Antioxidant activity	[157]
Skin	Theragra chalcogramma	Peptides	Protein-based secondary metabolites	Antioxidant activity	[158]
Gill and intestine	Morone saxatilis (stripped bass)	Peptide (Sb Piscidin 6)	Protein-based secondary metabolites	Antimicrobial	[137, 140]
Skin	Pterois volitans (lionfish)	Peptide (pteroicidin-*α* (-CONH_2_))	Protein-based secondary metabolites	Antimicrobial	[136, 137]
Scale	Oreochromis sp.	Collagen	Polysaccharide-based secondary metabolites	Tissue-engineered oral mucosa	[131, 132]
Cartilage	Prionace glauca, Zeachara chilensis, Bathyraja brachyurops	Collagen	Polysaccharides-based secondary metabolites	Bioscaffold	[141]
Skin	Paralichthys olivaceus	Collagen/polycaprolactone	Polysaccharides-based secondary metabolites	Bone regeneration	[131]
Scale	Ctenopharyngodon idella	Collagen	Polysaccharides-based secondary metabolites	Wound healing	[134]
Scale	Anabas testudineus	Chitosan	Polysaccharides-based secondary metabolites	Coagulation-flocculation treatment for iron removal	[135]
